The article "The Status Quo of College Students' Participation in English Online Learning in the Blended Learning Environment and the Ways to Improve It" was retracted in 2023. Reasons: signs of a paper mill; suspected computer-generated content; unreliable results or conclusions; lack of ethics approval or compliance.

# The Status Quo of College Students' Participation in English Online Learning in the Blended Learning Environment and the Ways to Improve It

**DOI:** 10.1155/2022/7255034

**Published:** 2022-08-12

**Authors:** Wanqi Cai

**Affiliations:** School of Education and Humanities, Xi'an Eurasia University, Xi'an 710065, Shaanxi, China

## Abstract

In college English teaching, online resources can meet students' self-study needs and show them a variety of English knowledge. Teachers should reasonably design teaching according to the characteristics of disciplines, and give students sufficient participation to conduct online self-study and online training. Therefore, online learning can make full use of students' spare time. In this paper, the current situation of college students' participation in online English learning and the ways to improve it are studied under the blended learning environment. The research shows that more than 88% of learners can finish online learning assignments on time. When the number of experiments reaches 60, 42.97% of them can finish online learning assignments on time, 29.51% of them can partially finish online learning assignments on time, and 21.94% of them cannot. In the process of online learning, autonomy and participation are high, and few of them are in a passive state, so they follow up online learning in time. The richness of college students' English online learning content under the blended learning environment provides a foundation, and college English teachers can optimize the learning content according to their lack of practical knowledge, which greatly improves college students' participation in online English learning.

## 1. Introduction

In the innovative development of college students' English teaching, teachers gradually pay attention to the application of online resources. With the help of information technology, we can improve the teaching atmosphere and make the English classroom full of vitality. In order to strengthen the English level of high school students and make information technology play a positive role in the English classroom, the hybrid teaching method should be used to guide students to carry out the in-class and after-class learning in an orderly manner, so as to improve the autonomy of learning participation, make teaching more scientific, and help students accumulate more English knowledge [1]. However, affected by the quality of online learning platform curriculum resources and students' participation in online courses, there is also great uncertainty in the new model of English online learning. Relevant scholars have found that the registration rate of online English learning is high, but the course completion rate is low, and that there are a lack of high-quality curriculum resources and the weakening of users' continuous participation in learning [2]. In University English teaching, online resources can meet students' self-study needs and show students a variety of English knowledge. Teachers should reasonably design teaching in combination with the characteristics of the subject, and give students sufficient participation in online self-study and online training. Therefore, online learning can make full use of students' spare time. At the same time, the practical knowledge of college students is practical, situational, personal, integrated, and reflective. The accumulation of practical knowledge of traditional college English teachers must be completed through teachers' practice and summary [3] and reasonably control the online and offline learning participation progress. Whether online or offline, students need to be given timely learning feedback. Carrying out some online tests based on online teaching platforms or other small programs is an important means to feedback students' learning effects. Through this feedback, we can make teaching activities more targeted, not only let students learn clearly, but also let teachers teach clearly. Of course, if we take the results of these small tests as an important basis for process evaluation, these test activities will also have the function of learning motivation. This mode can enrich students' learning content and training means, improve the efficiency of self-study after class, and promote learners' learning from shallow to deep to deep learning, which can not only improve English learning ability, but also have a positive impact on the learning of other disciplines.

In order to improve students' comprehensive quality and cultivate college students' participation in English online learning, we must first improve teachers' comprehensive quality, including professional quality. This paper analyzes the current situation of college students' participation in English online learning in a mixed learning environment and constructs a factor model for the continuous use of the college students' English online learning platform [4, 5]. By exploring the correlation between these influencing factors and college students' continuous use of online education platform, this paper puts forward corresponding improvement strategies for the University English online learning platform to adapt to the changes of college students' learning needs. Blended learning is a new learning mode that combines the advantages of various learning methods under the current educational informatization background. It mainly relies on traditional offline classroom learning and emerging online learning on network platforms. It can not only play the leading role of teachers' guidance, inspiration, and supervision in traditional classrooms, but also give students full learning autonomy. Blended learning, a combination of e-learning and traditional learning, has been widely spread and has become a hot topic in University English teaching reform. More and more universities gradually take blended learning as the basis of English learning, among which there are some stereotypes [6]. The actual implementation should be consistent, with blended learning as the core. However, due to poor equipment and related but defective facilities, policies and online learning cannot interact. Obviously, these have led to the failure of University English blended learning.

As a new learning mode, blended learning is more convenient and efficient, and brings students a sense of gain and satisfaction than other learning methods. At present, with more and more front-line teachers actively trying to carry out mixed teaching reform, the personalized learning needs of students in the mixed learning environment have been better met, and the students' autonomous participation in learning has also been further enhanced [7]. At the same time, teaching design should take learning as the center and students as the main information of the process, rather than following the continuous mode of students as passive recipients of stimuli from the outside [8]. Among many decisive factors, a successful methodology always serves the teaching goal. Specifically, how to design and conceive the correct learning program is really important. Therefore, the participation of college students in English online or distance education in blended learning means that students are actually far away from teachers and need a delivery method. The teacher-student interaction is determined by the design of technology and learning environment [9, 10]. The occurrence of spatial learning will have a considerable impact on the learning results. Online education has been studied for decades, and effective online teaching is the result of carefully designed and planned teaching. In addition, through the enrichment of college students' English online learning content in the hybrid learning environment, University English teachers can optimize the learning content according to their lack of practical knowledge, which greatly improves the participation of college students in English online learning.

For this paper, the following innovations are proposed:

1. A model of English online learning participation is proposed. Upload the teaching content to the “group file”; after class, the “homework” function is used to publish homework. Students can submit pictures, documents, and videos in various forms of homework. For common problems, the “micro class” function is used to explain them intensively, with good results. In order to avoid the tedium caused by teachers' single teaching in the teaching process, interactive content is added to the English online learning curriculum design. First of all, guide students to associate the real life that happens to them and around them with classroom learning, improve their divergent thinking ability, and enhance their learning initiative and enthusiasm.
2. This paper studies the application of blended learning in English online learning. Blended English teaching should be integrated into different links of English teaching. In the preview stage, teachers should formulate study plans to guide students to effectively self-study so that information technology can play a role and preview more efficiently. With the help of the advanced information technology, students can easily obtain extracurricular learning resources and listen to the pronunciation of vocabulary repeatedly, but they are prone to lack of direction due to too many resources.

The overall structure of this paper consists of five parts:

The first chapter introduces the background and significance of college students' English online learning and then introduces the main work of this paper. The second chapter mainly introduces the research status of English online learning and the research methods of English online learning proposed in this paper. The third chapter analyzes the research methods and discusses the participation in English online learning and the application of blended learning in English online learning. In Chapter 4, simulation experiments are carried out and the experimental results are analyzed. The fifth chapter is a summary of the full text.

## 2. Related Work

### 2.1. Research Status of Online English Learning

As there is an increase in the difficulty and the amount of knowledge, the review efficiency is particularly important. After the implementation of blended teaching, students can play a better role in autonomy, learn the content of micro-courses repeatedly, and have more and more vocabulary to use in dialogue. Therefore, it is necessary to continuously promote the integration of online and offline, and encourage students to improve their self-awareness. The after-class review and classroom teaching complement each other. Through self-questioning and self-reflection, the review objectives can be clearly defined, and the English level can be improved.

Gao et al. proposed that the stronger the compatibility of online education platform, the more reasonable the layout design of online education platform, the clearer the video images, and the better the audio quality, the more the college students who are willing to continue to use English online education platform for learning [11]. Kong proposed that the online education platform promoted by institution of higher learning will make full use of high-tech elements such as cloud technology and big data artificial intelligence to innovate online education mode and reshape learners' behavior. Particularly, the appearance of mobile terminal devices such as mobile phones and tablet computers has created sufficient conditions for online English learning in institution of higher learning. Therefore, online learning is supported and favored by many students [12]. Hu indicated that teachers should also integrate online and offline learning situations when making comments, and objectively evaluate students' learning attitudes and learning results so that students attach equal importance to online learning, and actively acquire learning resources to improve their learning autonomy [13]. Chen proposed that high-quality English teaching courses are the core of online learning platform service supply in institution of higher learning. If an online learning platform wants to run for a long time and maintain high popularity, it is essential for professional teachers to create high-quality and high-level English courses, so as to attract more learners and stimulate their willingness to continue online learning [14]. Truong and Wang showed there is a positive correlation between college students' feelings about the quality of English language teaching (ELT) content provided by an online platform and their willingness to continue using online platforms to learn English, and it is significant at the level of 0.01. Pearson's correlation coefficient is 0.745, which belongs to a strong correlation [15]. Liu et al. put forward that teachers should guide students to make self-evaluation, and find out the shortcomings of online English learning in combination with the teaching objectives of college students, so as to formulate a reasonable review plan and carry out an orderly review with the help of classroom notes and micro-course resources in the review stage. Many students cannot grasp the key points in the review, and they are used to reviewing from scratch according to the learning order, which leads to low review efficiency and weak grasp of important and difficult points [16]. Zhang showed that adding more real-time interactive means, such as online tutoring and online answering, can improve the interactivity of online English learning websites and systems. At the same time, various online activities should be provided for students to participate in, such as interactive games, competitions, and communities. Through timely feedback and real-time participation, students' learning initiative can be stimulated [17]. Chunlin et al. emphasized that the willingness to use continuously is the loyalty of college students' English learning users to the online education platform. Whether college students use online education platforms continuously or recommend each other actively can reflect the stickiness of the platform to users and the degree of college students' willingness to use continuously [18]. Chun meant to improve the intelligence of online English learning websites and systems and to strengthen the teaching assistance. In the process of developing websites and systems, we should give full consideration to how to give full play to teachers' guiding role and actively guide learners so that they can form a correct learning attitude and learning methods and establish a sound personality [19]. Liu et al. showed that college students who propose online English learning find that the more the students around them are also participating in online learning or the more the teachers and friends recommend them to use the online ELT platform, the more willing they are to continue to use the online ELT platform for learning [20].

### 2.2. The Research Method of English Online Learning Proposed in This Paper

Traditional classroom English teaching can no longer meet the increasing requirements of English learning, and the online English learning system provides a large number of constantly updated resources, breaks through the limitations of region and time, and provides students and teachers with an in-class or out-of-class online learning platform. In order to improve the effect of University English teachers' practical knowledge construction in online learning, it is necessary to effectively control the goal of college students' English online learning in the mixed learning environment in order to effectively control the participation in online learning. The generation of teachers' practical knowledge “emphasizes the overall perception, understanding, grasp, and processing of teaching situations by teachers in teaching activities.” Therefore, there are two important conditions for the generation of teachers' practical knowledge. First, there are problems in specific teaching situations. Second, there is reconstruction through reflection in action until new beliefs are formed. Teachers' practical knowledge is reflected in the process of problem-solving, and its formation environment is also inseparable from the specific education and teaching situation. Teachers, as professional practitioners, have a unique way of thinking, action, and teaching. Only when the education problem needs to be solved urgently, this kind of ability knowledge can be brought into play and developed. Reflection in action is the embodiment of the essential characteristics of this practical knowledge. Compared with the traditional offline classroom teaching, teachers have encountered unprecedented challenges. Some teachers have fallen far behind the pace of the times because they do not pay attention to these learning platforms and do not go to the library to borrow learning materials. It is necessary to build a hybrid learning oral English learning platform to ensure the development of online teaching. There are many network platforms. Choosing the appropriate teaching platform can effectively integrate resources and focus the attention of teachers and students on learning itself. University English teachers need to choose and use the functions and contents provided by the online learning platform in the process of online learning, not only to give full play to the value of the online learning environment, but also to curb the disadvantages of the online learning environment. Blended learning gives students with learning difficulties time to prepare before class, which is conducive to overcoming their fear of difficulties and learning difficulties; and gives students with good foundation and high requirements for oral English learning more difficult and diverse course choices to meet their requirements for continuous improvement. Therefore, if teachers do not learn and improve, and still adhere to the old and backward knowledge and teaching methods, teaching on the connection will become a problem, not to mention the teaching effect. Therefore, applying blended learning to college students' English online learning participation is the trend of future learning. Teachers must keep pace with the times and study modestly in order to cultivate more excellent college students.

## 3. Research Method

### 3.1. English Online Learning Participation

The theory of learning participation believes that learning participation reflects the level of time and energy invested by students in the learning process, which is divided into cognitive input, behavioral input, and emotional input. The higher the students' participation in learning, the higher the students' learning effect and development level, and the higher the educational quality level of institution of higher learning it reflects. There are many network platforms, so choosing a suitable English teaching platform can effectively integrate resources and focus the attention of teachers and students on learning itself [21, 22]. The teaching content is uploaded to the “group file”; after class, the “homework” function is used to publish homework. Students can submit pictures, documents, videos, and various forms of homework. For common problems, the “micro class” function is used to explain them intensively, with good results. In order to avoid the tedium caused by teachers' single teaching in the teaching process, interactive content is added to the English online learning curriculum design. First of all, the teachers guide students to associate the real life that happens to them and around them with classroom learning, improve their divergent thinking ability, and enhance their learning initiative and enthusiasm. English online teaching strategy has dynamic characteristics, including orientation strategy, interaction strategy, monitoring strategy, evaluation strategy, and feedback strategy, as shown in Figure 1.

The evaluation of learning participation has become an important index for the measurement and evaluation of educational quality in institution of higher learning, and has been paid more and more attention by educational administrators and front-line teachers in institution of higher learning. English online learning participation in the blended learning environment refers to the degree to which students participate in online courses synchronously or asynchronously using the online learning platform. It not only includes students' real-time participation in teachers' English online course teaching, but also includes students' self-study by logging on the English online learning platform after class [23]. The purpose of teaching strategy is to consciously monitor, evaluate, feedback, and adjust online teaching activities, coordinate the relationship between them as much as possible, optimize the teaching process, and achieve the teaching objectives more effectively. Therefore, the teaching strategy at this stage is not fixed, but it changes with the changes of learners, teaching context, teaching content, and other factors. It is necessary to carry out teaching activities according to the actual situation. It is particularly important to emphasize that at this stage, the single teaching link does not necessarily correspond to the teaching strategy of a teaching activity, but may also include guiding strategy, interactive strategy, and monitoring strategy [24]. On the basis of micro-courses and massive open online courses, building a flip classroom and giving students with learning difficulties preparation time before class will help them overcome their fear of difficulties and learning difficulties; giving students with good foundation and high English learning requirements more difficult and more diverse courses to choose will help them meet their requirements for continuous improvement.

In the process of online English teaching, multimedia materials such as words, pictures, videos, and audio are used, and a large number of interactive exercises, tests, thinking guidance, answering questions, and other activities are incorporated. Interactive design can play an active role in stimulating students' interest, timely feeding back the learning situation, achieving the test goal, activating students' thinking, etc., and help students better understand, absorb, and strengthen what they have learned [25]. All kinds of online English learning activities, such as autonomous learning, online questioning, online mutual evaluation, communication and discussion, homework completion, achievement sharing, and personal display, all reflect students' behavioral participation, emotional participation, and cognitive participation, which can truly and effectively reflect students' online English learning effect and personal development level [26].

### 3.2. The Application of Blended Learning in English Online Learning

Blended learning is a new concept put forward by the international educational technology community after in-depth consideration of networked learning based on the above understanding. A hybrid learning mode refers to a teaching method that fully integrates English online resources and offline teaching activities, gives full play to the advantages of information technology, guides students to explore independently, and effectively improves the teaching effect [27]. Blended English teaching should be implemented on the basis of mastering the discipline teaching rules. Teachers must reasonably plan English online and offline activities, guide students to learn new knowledge independently, use offline activities to test the results of self-study, and help students consolidate new knowledge and open their minds. Blended learning is a combination of online learning and face-to-face learning. It is necessary to adjust the effective mixing of learning elements such as various English learning media, learning modes, learning environment, and learning content, cultivate scholars' master learning ability, improve English learners' learning satisfaction, and optimize the combination of learning resources, so as to achieve the optimal learning effect and economic benefits. Online learning provides a learning environment with strong freedom for University English teachers, which highlights the dominant position of University English teachers in the construction of practical knowledge. However, if this freedom is not used properly, it will restrict the improvement of University English teachers' practical knowledge. In online learning, educators and learners, as well as learners and learners, are separated and do not have the binding and organizational atmosphere in the traditional classroom. Online learning can provide a platform for University English teachers to learn and communicate. University English teachers can enrich their practical knowledge according to the practice and experience of other teachers [28]. Of course, this kind of practical knowledge only includes practical knowledge that can be passed on and practical knowledge that can be understood. Some unconscious practical knowledge generated in teaching practice still needs teachers to summarize through English teaching practice.

However, blended learning should not be a simple mixture of two learning methods. Its core is to optimize the combination of learning resources according to the characteristics of the subject and make scientific and reasonable use of English resources. At present, the research on blended English learning in the foreign language community is not systematic enough. It mostly focuses on the simple combination of network and classroom English teaching mode, and has little guiding significance for teachers to carry out blended teaching. There are few studies on the integration of learning and classroom English teaching, teacher-student interaction, evaluation and feedback based on educational technology, and student-centered and comprehensive improvement of students' English professional ability. The optimization of the University English teachers' online learning environment focuses on optimizing the online learning platform composed of the Internet and computer, so as to make the online learning environment meet the needs of University English teachers' practical knowledge development; that is, it is required that the online learning environment should conform to the cognitive law of University English teachers' practical knowledge after optimization. Combining the traditional face-to-face classroom teaching method with the online autonomous learning method, turning the classroom, and learning through online and offline not only give play to the leading role of teachers, but also highlight the central position of learners through platform learning and cultivate learners' autonomous learning ability. The structure of the hybrid learning space is shown in Figure 2.

Blended English teaching should be integrated into different links of English teaching. In the preview stage, teachers should formulate learning plans, guide students to learn by themselves effectively, make information technology play a role, and make the preview more efficient. With the help of the advanced information technology, students can easily get extracurricular learning resources and listen to the pronunciation of vocabulary repeatedly, but it is easy to lack directionality due to too many resources. Because there are too many links in the online learning platform and college English teachers' attention is distracted, college English teachers who lack solid English professional knowledge and teaching ability will have double learning pressure brought by practical knowledge and computer operation knowledge, and the openness of learning, that is, learning content, all of which require college English teachers to make independent choices to prevent English teachers from having negative attitudes towards learning content. Self-regulated learning in the online learning environment and cooperative learning in a classroom learning environment combine and complement each other, so as to construct a brand-new learning method that can not only play the leading role of classroom learning teachers, but also embody students' knowledge construction through English learning. Rich network resources can make up for the shortage of high-quality resources in local universities.

The blended English online learning platform can provide students with all kinds of English teaching materials related to courses, such as open classes in famous universities, micro-classes, PPT in classroom teaching, supplementary materials, and links to references. The mixing of conventional classroom teaching platforms, combined with the concept of a flipped classroom, reflects the multidimensional collaborative thinking of both inside and outside the classroom, online and offline, knowledge and skills, and equal emphasis on teaching and acquisition. It is the fusion of the essence of the traditional teaching mode and the modern educational technology, and the service quality of the online platform and the influence of the students' user community. Therefore, the improvement strategies to enhance college students' willingness to use English online education platform should also be considered around these four factors.

## 4. Result Analysis and Discussion

This empirical study uses the reliability coefficient method to test the internal reliability of the option questionnaire. The value of the Cronbach coefficient method is used as the benchmark to measure the reliability. The higher the coefficient is, the more consistent the monitoring results are and the more reliable the data are. In specific research, the measurement items with a reliability coefficient of more than 0.7 are usually judged to have good stability. The reliability measurement results of the questionnaire data of this sampling survey are shown in Table 1.

The Cronbach coefficient a value of each variable is greater than 0.7, indicating that the data are stable and the survey has good reliability. The teacher-student interaction is an important way of communication between teachers and students in the modern education system, and it is an important influencing factor for the smooth development of teaching, especially in the mixed learning mode. The teacher-student interaction is divided into two levels: the interaction between teachers and students and the interaction between students and students. The investigation is carried out to clarify the current situation and improve the deficiencies. This experiment mainly carries out experimental analysis from three categories: I like teachers to give feedback in time; I like to ask questions directly from teachers face-to-face; and I like to ask questions from teachers through the Internet, and then I analyze complete nonconformity, partial conformity, and complete conformity. The statistical analysis results of the teacher-student interaction are shown in Figure 3.

66% of learners prefer to ask questions through the Internet. The data show that learners prefer to communicate with teachers through the Internet under the blended learning mode, which is in line with the characteristics of the contemporary era. Only 12% of learners do not agree with the questions that teachers like to give feedback in time, which indicates that in the process of the teacher-student interaction, teachers should pay attention to timely feedback information to students, and guide them to learn efficiently and actively. Accurate feedback is the direction and motivation of learners' learning.

The frequency of each online English teaching strategy is counted in the teaching stage, as shown in Table 2, and the frequency ratio data after the frequency statistics are summarized. Through these frequency data, the use and characteristics of teachers' teaching strategies can be calculated more intuitively.

In the survey of self-cognition, most learners also have a clear level of self-cognition. Therefore, in order to improve learners' dominant position, self-evaluation and peer evaluation can also be included in the evaluation index system. Therefore, this experiment is aimed at completely inconsistent, partially consistent, and completely consistent learning. Blended learning pays more attention to learning process experience. Learning experience is the effect of learners' experience in the learning process, as shown in Figure 4.

More than 82% of learners hold a positive attitude and positive emotional experience towards the blended learning model, and it can be seen that full compliance accounts for the highest proportion in the process of blended learning, followed by partial compliance, and finally completely noncompliance. They recognize the hybrid learning method and pay attention to the learning process; from the perspective of learners' after-school learning, most learners like to reflect and summarize what they have learned, thought, and realized. In the process of English evaluation methods, we can appropriately add evaluation methods that meet the learners' self-improvement psychology, pay attention to the learners' progress in the learning process, and give feedback and evaluation in time, so as to increase learners' confidence, improve learning experience and satisfaction, and study efficiently.

Online learning participation refers to the degree to which learners participate in online learning under the hybrid learning mode, mainly from the learners' attitude towards online learning, time, number of login platforms, and resource sharing. This experiment aims at completely nonconforming, partially conforming, and fully conforming learning. The experiment is carried out to complete the online learning homework on time. The experimental results are shown in Figure 5.

More than 88% of learners can complete online learning assignments on time. As can be seen from the figure, when the number of experiments reaches 60, 42.97% of them are fully qualified to complete online learning assignments on time, 29.51% are partially qualified to complete online learning assignments on time, and 21.94% are completely unqualified to complete online learning assignments on time. In the process of online learning, autonomy and participation are high, and a few are in a passive state. It can be seen that most learners have a correct attitude towards online learning, recognize online learning methods, and follow up online learning in time. In the evaluation system, we can properly consider the learner's autonomy factors, pay attention to the learner's learning process, such as the number of forum discussions and online tests, and incorporate the corresponding evaluation methods to improve the enthusiasm of learners.

As for the question “what kind of learning method do you want to use if there are bilingual teaching courses in the future” in our interview, almost all the students who participated in the interview answered “blended learning.” It can be seen that the role of blended learning in bilingual teaching has left a deep impression on students. Therefore, this experiment aims at the improvement of learners' ability. Three methods are adopted for comparison, namely, machine learning, ant colony algorithm, and hybrid learning in this paper. The experimental results are shown in Figure 6.

From the data of the three methods, it can be seen that the growth value of blended learning in this method is the highest, followed by ant colony algorithm, and finally by machine learning. Therefore, it can be concluded that blended learning can make learners gain a lot, and students think that blended learning improves their information literacy; some learners think that blended learning helps them master knowledge; others think that blended learning improves their skills and practical ability; and others think that they improve their computer ability. According to the correlation analysis between college students' willingness to use continuously and various factors, see Table 3.

College students' perception of service quality of online platform is positively correlated with their willingness to continue to use online platform to learn English, and it is significant at the level of 0.02. Pearson's correlation coefficient is 0.622, which is a strong correlation. At the same time, there is a significant correlation between college students' willingness to use continuously and the service quality of college English online platform.

Blended learning improves English listening and reading. On the learning platform, we uploaded a large number of reading materials and video materials according to the course content, and learners unconsciously improved their English listening and reading ability while learning professional knowledge. In this experiment, aiming at English ability, the category has been greatly improved, and it has been improved to a certain extent. The experimental analysis has been carried out without any improvement, and the experimental results are shown in Figure 7.

Among the three categories, a certain increase is the highest in the three growth rates, with an average growth rate of 29.19%. In the second place, there was a great improvement, with an average growth rate of 21.75%. Finally, there was no improvement, with an average growth rate of 14.24%. Because we have added more cutting-edge knowledge of the discipline to the expanded resources, including the speech videos of some foreign experts and excellent research papers, students can read these expanded resources and record their learning experiences after learning the classroom knowledge. Through these exercises, students have more understanding of the cutting-edge knowledge of the discipline, thus expanding their professional vision.

## 5. Conclusions

University English online learning adopts the way of physical incentives to encourage learning participants to share their online learning experience with various social platforms on campus in a variety of ways, so as to achieve the purpose of effective publicity of positive word of mouth. This is also an important way to use community influence to promote college students' online learning. This paper studies the current situation and improvement path of college students' English online learning participation in a hybrid learning environment. The research shows that more than 88% of learners can complete online learning assignments on time. When the number of experiments reaches 60, 42.97% of them are fully qualified to complete online learning assignments on time, and 29.51% of them are partially qualified to complete online learning assignments on time, 21.94% did not meet the requirements of completing online learning assignments on time. In the process of online learning, autonomy and participation are high, and a few are in a passive state. It can be seen that most learners have a correct attitude towards online learning, recognize online learning methods, and follow up online learning in time. The scientific and reasonable use of hybrid learning evaluation can monitor the dynamic learning process of learners, exercise learners' autonomy, initiative, and innovation, master learning skills, improve learning quality, and develop themselves in an all-round way; at the same time, it can guide teachers to reasonably arrange teaching progress and arrangement, do a good job of teaching adjustment at any time, improve teaching level, promote the harmonious development of teacher-student relationship, and improve the participatory evaluation method system.

## Figures and Tables

**Figure 1:** English online learning participation model.

**Figure 2:** Student-centered blended learning space.

**Figure 3:** Statistical analysis of the interaction between teachers and students.

**Figure 4:** Blended learning pays more attention to the change of learning experience in the learning process.

**Figure 5:** Change trend of being able to complete online learning assignments on time.

**Figure 6:** Curve of improvement of learners' ability under different methods.

**Figure 7:** Improvement of English ability.

**Table 1:** Reliability coefficients of variables in empirical research.

Variable name	Cronbach's coefficient a value	Cronbach's coefficient a value based on standardization term
Performance expectations	0.896	0.934
Service quality	0.921	0.953
Willingness to continue using	0.892	0.896
Social influence	0.982	0.911

**Table 2:** Statistical table of the usage of teaching strategies in the teaching stage.

While-teaching stage					
Observation indicators	Guidance strategy	Interaction strategy	Monitoring strategy	Evaluation strategy	Feedback strategy
Lead in	82%	66.8%	6.8%	33.4%	0%
Development	26.6%	26.8%	41%	13.4%	33.4%
Presentation	86.8%	66.8%	26.8%	13.4%	21%
Total	68.7%	54.4%	52.5%	41.2%	41.2%

**Table 3:** Correlation analysis between college students' willingness to use English online education platform and various factors.

Variable	Pearson's correlation coefficient	Significant bilateral test
Performance expectation	0.622	0.000
Quality of service	0.744	0.000
Willingness to use continuously	0.682	0.000
Community influence	0.872	0.000

## Data Availability

The figures and tables used to support the findings of this study are included in the article.
